# Induction of metastasis, cancer stem cell phenotype, and oncogenic metabolism in cancer cells by ionizing radiation

**DOI:** 10.1186/s12943-016-0577-4

**Published:** 2017-01-30

**Authors:** Su Yeon Lee, Eui Kyong Jeong, Min Kyung Ju, Hyun Min Jeon, Min Young Kim, Cho Hee Kim, Hye Gyeong Park, Song Iy Han, Ho Sung Kang

**Affiliations:** 1 Department of Molecular Biology, College of Natural Sciences, Pusan National University, Pusan, 609-735 Korea; 2 Research Center, Dongnam Institute of Radiological and Medical Science (DIRAMS), Pusan, 619-953 Korea; 3 DNA Identification Center, National Forensic Service, Seoul, 158-707 Korea; 4 Nanobiotechnology Center, Pusan National University, Pusan, 609-735 Korea; 5 The Division of Natural Medical Sciences, College of Health Science, Chosun University, Gwangju, 501-759 Korea

**Keywords:** Radiotherapy, Epithelial-mesenchymal transition, Metastasis, Cancer stem cells, Oncogenic metabolism, Tumour microenvironment, Reactive oxygen species, Radioresistance, Snail

## Abstract

Radiation therapy is one of the major tools of cancer treatment, and is widely used for a variety of malignant tumours. Radiotherapy causes DNA damage directly by ionization or indirectly via the generation of reactive oxygen species (ROS), thereby destroying cancer cells. However, ionizing radiation (IR) paradoxically promotes metastasis and invasion of cancer cells by inducing the epithelial-mesenchymal transition (EMT). Metastasis is a major obstacle to successful cancer therapy, and is closely linked to the rates of morbidity and mortality of many cancers. ROS have been shown to play important roles in mediating the biological effects of IR. ROS have been implicated in IR-induced EMT, via activation of several EMT transcription factors—including Snail, HIF-1, ZEB1, and STAT3—that are activated by signalling pathways, including those of TGF-β, Wnt, Hedgehog, Notch, G-CSF, EGFR/PI3K/Akt, and MAPK. Cancer cells that undergo EMT have been shown to acquire stemness and undergo metabolic changes, although these points are debated. IR is known to induce cancer stem cell (CSC) properties, including dedifferentiation and self-renewal, and to promote oncogenic metabolism by activating these EMT-inducing pathways. Much accumulated evidence has shown that metabolic alterations in cancer cells are closely associated with the EMT and CSC phenotypes; specifically, the IR-induced oncogenic metabolism seems to be required for acquisition of the EMT and CSC phenotypes. IR can also elicit various changes in the tumour microenvironment (TME) that may affect invasion and metastasis. EMT, CSC, and oncogenic metabolism are involved in radioresistance; targeting them may improve the efficacy of radiotherapy, preventing tumour recurrence and metastasis. This study focuses on the molecular mechanisms of IR-induced EMT, CSCs, oncogenic metabolism, and alterations in the TME. We discuss how IR-induced EMT/CSC/oncogenic metabolism may promote resistance to radiotherapy; we also review efforts to develop therapeutic approaches to eliminate these IR-induced adverse effects.

## Background

Ionizing radiation (IR) is an effective and common therapeutic tool for cancer treatment. More than half of cancer patients are treated with IR at some point during their treatment, either alone or in combination with surgery and/or chemotherapy [1–6]. In radiotherapy, fractionated treatment regimens have been established. The standard fractionation schedule is the delivery of 1.8–2.0 Gy per day, five days per week. This reduces side effects, and allows damaged normal cells to recover before additional doses are given [4, 5]. Fractionated radiotherapy increases damage to the tumour; it may reoxygenate the tumour cells and re-distribute their cell cycles into more sensitive phases. It also minimises repopulation of the tumour during therapy [2, 4, 7].

Nuclear DNA is the primary target of IR; it causes DNA damage (genotoxic stress) by direct DNA ionization. IR also indirectly induces DNA damage by stimulating reactive oxygen species (ROS) production [8–15]. The therapeutic effects of IR are traditionally associated with the DNA double-strand breaks (DSBs) that are the most lethal form of damage to tumour cells. Much evidence has shown that p53 is activated in response to IR-induced DNA damage [8–11]. p53 is a multifunctional transcription factor and it acts principally as a tumour suppressor. It increases the expression of several genes to induce cell cycle arrest (p21, 14-3-3σ), apoptosis (PUMA, NOXA, BAX), autophagy (phosphatase and tensin homolog [PTEN], TSC1, DRAM), or senescence (p21), depending on the cell type and the severity of damage [9, 10]. These are important therapeutic effects of IR.

ROS have been shown to play an important role in mediating the biological effects of IR [12–19]. IR can increase ROS production both by inducing extracellular water radiolysis and by causing intracellular metabolic changes or damage to mitochondria. IR induces delayed (24 h onward), persistent (for days) increases in mitochondrial ROS production, while ROS generated from water have very short life spans (10^-9^ s) [15, 17]. IR also induces a reversible mitochondrial permeability transition that stimulates ROS production [16]. IR-induced mitochondrial ROS production is associated with partial deactivation of mitochondrial respiratory complexes I and III of the electron transport chain [18, 19]. In turn, excess ROS can disrupt intracellular oxidation/reduction systems and cause oxidative damage to biomolecules, including DNA [12–15]. Activation of the mitochondrial permeability transition also increases levels of reactive nitrogen species (RNS), such as nitric oxide (NO) [16].

Although IR is used as a standard treatment for a variety of malignant tumours, IR paradoxically also promotes tumour recurrence and metastasis [20–28]. The epithelial-mesenchymal transition (EMT) has been shown to endow cancer cells with migratory and invasive properties, enabling the initiation of metastasis [29–31]. IR is known to induce EMT in vitro [20–26]. EMT may be closely linked to cancer stem cells (CSCs) and the metabolic reprogramming of cancer cells, although there is disagreement in the field on these points.

IR is known to induce stemness and metabolic alterations in cancer cells; IR can also cause various changes in the tumour microenvironment (TME) that may promote tumour invasion and metastasis. Oncogenic metabolism has been shown to play important roles in the acquisition of EMT and CSC phenotypes; thus, IR seems to induce EMT and CSC phenotypes by regulating cellular metabolism. EMT, stemness, and oncogenic metabolism are known to be associated with resistance to radiotherapy and chemotherapy. Therefore, understanding the molecular mechanisms of IR-induced EMT/CSC/oncogenic metabolism and changes in the TME is required to improve the efficacy of radiotherapy. Here, we review recent advances in the understanding of the molecular mechanisms of IR-induced EMT, CSC, oncogenic metabolism, and changes in TME, and we discuss a relationship between EMT/CSC/oncogenic metabolism and radioresistance.

### Induction of EMT, invasion, and metastasis by IR

#### EMT, invasion, and metastasis

Cancer cells can acquire multiple biological capabilities during their multistage development. Hanahan and Weinberg proposed ten hallmarks of cancer that alter cell physiology to enhance malignant growth: 1) sustained proliferation, 2) evasion of growth suppression, 3) cell death resistance, 4) replicative immortality, 5) evasion of immune destruction, 6) tumour-promoting inflammation, 7) activation of invasion and metastasis, 8) induction of angiogenesis, 9) genome instability, and 10) alteration of metabolism [32, 33]. Recently, it has also been suggested that cancer is characterised by a breakdown of multicellular cooperation by instances of cellular “cheating” that disrupt all of the following: proliferation inhibition, regulation of cell death, division of labour, resource transport, and maintenance of the extracellular environment. Furthermore, it has also been suggested that deregulation of differentiation is another important aspect of tumourigenesis [34] (Fig. 1).

**Fig. 1:** Epithelial-mesenchymal transition (EMT), metastasis, cancer stem cells (CSCs), and oncogenic metabolism. Cancer cells can acquire multiple capabilities, including sustained proliferation, evasion of growth suppression, cell death resistance, replicative immortality, evasion of immune destruction, tumour-promoting inflammation, activation of invasion and metastasis, induction of angiogenesis, genome instability, and alteration of metabolism. Deregulation of differentiation, acquisition of stem cell phenotypes, and their tumour microenvironment are also important aspects of tumourigenesis. Several signal pathways (such as those of TGF-β, Wnt, EGF, Hedgehog, Notch, and ROS) and mutation/genomic instability are closely associated with tumourigenesis and tumour progression. These signals could activate oncogenes and inactivate tumour suppressors. Activation of oncogenes, or loss of tumour suppressors, can drive tumour progression, particularly via metabolic reprogramming. Metabolic reprogramming may be required for malignant transformation and tumour development, including invasion and metastasis, CSC phenotype, and TME

Among the known characteristics of cancer, metastasis is the major obstacle to therapeutic access [29, 35, 36]. EMT is closely linked to the induction of metastasis. EMT is a developmental process that plays critical roles in embryogenesis, wound healing, and organ fibrosis [29–31]. EMT confers mesenchymal properties on epithelial cells; it is characterised by the loss of epithelial morphology and markers (including E-cadherin, desmoplakin, Muc-1, cytokeratin-18, occludins, claudins, and ZO-1), and by the acquisition of mesenchymal markers (including N-cadherin, vimentin, fibronectin, vitronectin, α-smooth muscle actin [α-SMA], and FSP1). Thus, cancer cells undergoing EMT acquire invasive and metastatic properties [29–31].

EMT programs are regulated by a network of signalling pathways that involve components such as growth factors (transforming growth factor-β [TGF-β], epidermal growth factor [EGF]) and their associated signalling proteins (Wnt, Notch, Hedgehog, nuclear-factor kappa B [NF-κB], extracellular signal-regulated kinase [ERK], and phosphatidylinositol 3-kinase [PI3K]/Akt) in response to stresses involved in tumourigenesis, including hypoxia, oncogenic or metabolic stress, inflammation, and physical constraints [30, 31, 37–39].

These signals activate EMT-inducing transcription factors, including Snail/Slug, ZEB1/δEF1, ZEB2/SIP1, Twist1/2, and E12/E47 [40–42]. EMT-inducing transcription factors regulate the expression of proteins involved in cell polarity, cell-cell contact, cytoskeletal structural maintenance, and extracellular matrix (ECM) degradation, and they suppress key epithelial genes. Loss of E-cadherin is considered a hallmark of EMT; these EMT-inducing transcription factors bind to E-box elements in the E-cadherin gene promoter to repress its transcription. Of particular note, Snail is an early marker of EMT that is involved in the initial cell-migratory phenotype, and it occasionally induces other factors [40–42].

In addition to having pro-metastatic roles, these EMT-inducing transcription factors are also implicated in tumour initiation and early tumour development. Their oncogenic potential has proven to be associated with the capacity to inhibit tumour-suppressive 'fail-safe' programs (senescence and apoptosis), and to induce stemness properties and metabolic alterations. The Twist protein is known to inhibit senescence and apoptosis. Although the roles of Snail and ZEB in senescence are debated, these proteins have been shown to confer resistance to cell death. Snail, ZEB, and Twist also induce malignant transformation, as well as the acquisition of stemness properties [40, 43]. Emerging evidence also shows that Snail can promote metabolic alterations [42, 43]. The roles of these proteins in the CSC phenotype, metabolic alteration, and resistance to therapy will be addressed in more detail below.

#### Induction of EMT, invasion, and metastasis by IR

IR has been shown to induce EMT to enhance the motility and invasiveness of several cancer cells, including those of breast, lung, and liver cancer, and glioma cells [20–27]. Clinical and preclinical evidence suggests that IR may increase metastasis in both the primary tumour site and in normal tissues under some circumstances [20, 23, 27]. Even sublethal doses of IR have been shown to enhance the migratory and invasive behaviours of glioma cells [21, 22].

ROS are known to play an important role in IR-induced EMT [44, 45]. ROS act as second messengers in intracellular signalling that induce tumourigenicity and sustain tumour progression. ROS have been closely associated with tumourigenesis and tumour progression. ROS can act as signalling molecules that regulate cell proliferation and death [46–52]. Mitochondrial ROS production is known to be activated by hypoxia, oncogenes, loss of tumour suppressors, or mitochondrial mutations to increase tumourigenicity [50, 51]. High levels of ROS trigger cell death by causing irreversible damage to cellular components such as proteins, nucleic acids, and lipids, whereas low levels of ROS have been shown to promote tumour progression—including tumour growth, invasion, and metastasis [46–52]. It has been noted that cancer cells also express high levels of antioxidant proteins to inhibit ROS-induced cytotoxicity [47–49, 51]. Therefore, ROS levels are crucial for radiotherapy outcomes. ROS promote EMT to allow cancer cells to avoid hostile environments [46–49, 52].

IR can induce ROS production directly and indirectly, by extracellular water radiolysis and by intracellular metabolic alterations or mitochondrial dysfunction [15, 17]. Treatment with the N-acetylcysteine (NAC), a general ROS scavenger, prevents IR-induced EMT, adhesive affinity, and invasion of breast cancer cells, suggesting an important role for ROS in IR-induced EMT [44, 45].

Snail has been shown to play a crucial role in IR-induced EMT, migration, and invasion [53–56]. ROS are also involved in IR-induced Snail expression. IR-induced ROS activate ERK1/2, which inactivates glycogen synthase kinase 3β (GSK3β), an endogenous inhibitor of Snail, thereby upregulating Snail [53]. Sustained elevation of Snail expression is required for IR-induced ERK activation and GSK3β inhibition, suggesting that ERK/GSK3β/Snail might form a positive feedback loop [54]. Several signalling pathways have also been implicated in IR-induced Snail expression, including TGF-β, Wnt, Hedgehog, Notch, granulocyte-colony stimulating factor (G-CSF), EGFR/PI3K/Akt, mitogen-activated protein kinase (MAPK), and p21-activated kinase 1 (PAK1), as discussed below. IR activates the p38 MAPK pathway, which contributes to the induction of Snail expression to promote EMT and invasion [56]. PAK1 is also activated by IR, after which it directly binds to Snail, which increases the transcriptional repression activity of Snail, thereby repressing E-cadherin expression [55].

Snail is known to be regulated by distal-less homeobox-2 (Dlx-2) [57, 58]. Dlx-2 is a homeobox transcription factor and is involved in embryonic and tumour development [59–63]. We previously showed that Dlx-2 acts as an upstream regulator of Snail [57, 58]. In addition, IR has been shown to upregulate Dlx-2 by activating Smad2/3 signalling that induces EMT in A549 and MDA-MB-231 cell lines [64]. We also found that Dlx-2 is implicated in IR-induced EMT by activating Snail; Dlx-2 expression was increased by IR-induced ROS. Dlx-2 shRNA suppressed the IR-induced EMT phenotype, and was accompanied by downregulation of Snail (data not shown; see the abstract of MSIP reports (No. 2012M2B2A9A02029802; http://www.ndsl.kr/ndsl/search/detail/report/reportSearchResultDetail.do?cn=TRKO201300032641 and No. 2013M2B2A9A03050902; http://www.ndsl.kr/ndsl/search/detail/report/reportSearchResultDetail.do?cn=TRKO201600009259). These results suggest that IR induces EMT via ROS-dependent activation of Dlx-2 and Snail.

In addition, ultraviolet (UV) radiation, a form of non-IR, which is considered the main cause of skin cancer, is also known to enhance cell migration by increasing ROS levels, similar to IR. UV radiation-induced ROS activates NF-κB signalling that promotes cell migration [65]. NF-κB is known to increase Snail stabilisation by preventing the ubiquitination and degradation of Snail, which promotes cell migration and invasion [66, 67]. Snail also plays an important role in UV radiation-induced EMT. UV radiation induces Snail expression by activating the EGFR, ERK, and p38 MAPK cascades [68–70]. MAPK signalling activates AP-1 transcription factor to directly increase Snail expression in keratinocytes [69].

ZEB1 is also implicated in IR-induced EMT [71, 72]. IR-induced GSK3β inactivation has been shown to contribute to the induction of ZEB1 expression [72]. IR also promotes Akt phosphorylation to elevate ZEB1 expression, which promotes EMT. Indeed, following radiotherapy, high levels of ZEB1 and phosphorylated Akt (S473) are correlated with recurrence and distance metastasis in patients with nasopharyngeal carcinoma [71].

In addition, hypoxia-inducible factor-1 (HIF-1) is involved in IR-induced EMT [73–82]. HIF-1 is a heterodimer composed of an oxygen-sensitive α subunit and a constitutively expressed β subunit. Under normoxia, HIF-1α is rapidly degraded, whereas hypoxia induces stabilisation and accumulation of HIF-1α [73–76]. Several mechanisms are known to induce HIF-1 activation by increasing the translation of HIF-1α mRNA or inhibiting HIF-1α degradation; levels of HIF-1α mRNA are enhanced by activation of the PI3K/Akt/mammalian target of rapamycin (mTOR) pathway and by the binding of YB-1, an RNA and DNA binding protein. HIF-1α protein degradation has been prevented by ROS and NO. Inactivation of von Hippel-Lindau tumour suppressor protein (pVHL, an E3 ubiquitin ligase targeting HIF-1α) and activation of WSB1 (an E3 ligase targeting pVHL) and ubiquitin C-terminal hydrolase-L1 (UCHL1, a HIF-1 deubiquitinating enzyme) are also known to induce HIF-1α stabilisation and activation [73–77].

IR is known to increase stabilisation and nuclear accumulation of HIF-1α, since hypoxia is a major condition for HIF-1 activation [73, 75]. IR induces vascular damage that causes hypoxia. In addition, ROS is implicated in IR-induced HIF-1 activation; IR causes the reoxygenation of hypoxic cancer cells to increase ROS production, which leads to the stabilisation and nuclear accumulation of HIF-1 [77, 78]. IR-induced reoxygenation also enhances the translation of HIF-1-regulated transcripts [77]. In addition, IR increases glucose availability under reoxygenated conditions that promote HIF-1α translation by activating the Akt/mTOR pathway [78]. Furthermore, IR upregulates Nijmegen breakage syndrome protein 1 (NBS1), which directly interacts with HIF-1α and stabilises it [80]. The stabilised HIF-1α then translocates to the nucleus, dimerizes with HIF-1β, and increases gene expression— including the expression of essential EMT regulators such as Snail—to induce EMT, migration, and invasion [73, 83].

A number of signalling pathways, including those of TGF-β, Wnt, Hedgehog, Notch, G-CSF, EGFR/PI3K/Akt, CXCL12/CXCR4, PAI-1, and MAPK, have been implicated in IR-induced EMT [45, 84–117] (Fig. 2). TGF-β signalling has been shown to play a crucial role in IR-induced EMT [84–94]. Among three isoforms of TGF-β (TGF-β1, TGF-β2, and TGF-β3), IR is known to specifically induce TGF-β1 [84, 85]. AP-1 transcription factor is involved in IR-induced TGF-β1 expression [84]. After it is synthesised, TGF-β is secreted as an inactive homodimer that binds to latent TGF-β binding protein (LTBP), forming a latent complex. The latent TGF-β complexes can be activated by extracellular stimuli (ROS and acidic conditions) or by the proteolytic activity of proteases (matrix metalloproteinase [MMP]-2 and MMP-9) [87, 88].

**Fig. 2:** Signalling pathways of IR-induced EMT, metastasis, CSCs, and oncogenic metabolism. Ionizing radiation (IR) causes DNA damage directly, by ionization, or indirectly, by the production of reactive oxygen species (ROS) in tumours. In response to DNA damage, p53 is activated and it exerts the therapeutic effects of IR: induction of cell cycle arrest, apoptosis, autophagy, or senescence. However, IR is also known to enhance the metastatic potential of cancer cells by inducing EMT. IR-induced EMT is mediated by transcription factors (including Snail, HIF-1, ZEB1, Twist, and STAT3) that are activated by signalling pathways (including those of TGF-β, Wnt, Hedgehog, Notch, G-CSF, EGFR/PI3K/Akt, CXCL12/CXCR4, PAI-1, and MAPK). ROS are implicated in IR-induced EMT via the activation of these transcription factors and signalling pathways. Cancer cells that undergo EMT also acquire stemness and oncogenic metabolisms. In addition, EMT, CSCs, and oncogenic metabolism are known to contribute to the radioresistance of cancer cells

IR-induced ROS is known to promote the extracellular proteolytic cleavage of latent complexes so that the biologically activated TGF-β can bind to its receptors [86]. TGF-β binds with the TGF-β type II receptor (TβRII); this receptor-ligand complex recruits and phosphorylates a TGF-β type I receptor, ALK5. ALK5 then phosphorylates the proteins Smad2 and 3, which bind to Smad4 and translocate to the nucleus, where they transactivate target genes [87, 88]. In addition to activation of the synthesis and secretion of TGF-β1, IR promotes intracellular TGF-β signalling, as evidenced by the phosphorylation of Smad 2/3C and the upregulation of its target genes (TβRII and ALK5), thereby leading to hyperactivation of TGF-β signalling [93]. Furthermore, IR elevates FoxM1, which acts downstream of TGF-β1/Smad signalling. IR-induced FoxM1 directly binds to the Snail promoter and increases Snail expression to mediate TGF-β-induced EMT [92].

Wnt/β-catenin signalling is also implicated in IR-induced EMT [95–98]. IR has been shown to increases Wnt signalling by increasing Wnt ligand expression [96]. Generally, Wnt binds to its receptor Frizzled and to its co-receptor, lipoprotein receptor-related protein (LRP) 5/6 that suppresses GSK3β-mediated phosphorylation of β-catenin [39]. IR is known to enhance β-catenin stabilisation [95, 97]. Subsequently, the stabilised β-catenin is translocated to the nucleus and binds to T-cell factor (TCF)/lymphoid enhancer factor (LEF) transcription factors to activate target gene expression [39]. IR also induces the nuclear translocation and accumulation of β-catenin, and increases β-catenin/TCF transcriptional activities [95, 98].

In addition, Wnt signalling increases Snail protein stability in the nucleus by activating an Axin2 pathway, thereby inducing EMT. Axin2 acts as a chaperone for nuclear export of GSK3β, the dominant kinase responsible for Snail protein turnover and activity [118, 119]. Recently, we showed that the Dlx-2/Snail cascade is implicated in TGF-β- and Wnt3a-induced EMT [57]. IR-induced Wnt/β-catenin signalling elevates Snail to promote EMT, migration, and invasiveness of progeny from irradiated colorectal cancer cells [95, 97].

Notch signalling is known to be involved in IR-induced EMT [99, 100]. Notch signalling is activated by interaction between transmembrane Notch receptors (Notch 1–4) and ligands (Jagged-1, Jagged-2, Delta-like 1, Delta-like 3, Delta-like 4) on contacting cells. IR activates the IL-6/JAK/signal transducer and activator of transcription 3 (STAT3) pathway to upregulate Notch-2, Jagged1, and Delta-like 4, and induces EMT [100]. IR also increases Notch-1 expression [99]. Notch-1 is known to induce EMT by upregulating Snail. Treatment with two Notch-1-regulating radiosensitizers, rhamnetin and cirsiliol, induces the miR-34a-mediated downregulation of Notch-1, preventing IR-induced EMT [99].

IR has also been shown to activate Hedgehog (Hh) signalling to induce EMT [101]. IR increases expression of the Hh ligand (Indian Hh, Sonic Hh), the Hh receptor (Smoothened), and the Hh-target gene (Gli2), with enhanced expression of the EMT-stimulating factor (TGF-β) and mesenchymal markers (N-cadherin, α-SMA). Blocking Hh activity suppresses the IR-induced expression of EMT-stimulating genes, suggesting a potential role for Hh signalling in IR-induced EMT [101].

Furthermore, EGFR activation is known to be associated with IR-induced EMT, cell migration, and invasion by activating two downstream pathways: PI3K/Akt and Raf/MEK/ERK [45, 102–108]. Ligand binding to EGFR generally induces receptor dimerization, activation of its kinase domain, and consequent autophosphorylation [102, 103]. IR promotes EGFR heterodimerization with ErbB2 in a ligand-independent manner [104].

ROS and RNS are also implicated in IR-induced EGFR activation [45, 105]. IR-induced ROS are known to promote phosphorylation of EGFR or ErbB2 Y^877^ [45, 105]. IR-induced RNS also induce autophosphorylation on EGFR Y^1173^. Following IR, NO is generated within minutes, which is necessary for the rapid activation of EGFR [105]. UV-induced ROS are also implicated in IR-induced EGFR activation. NAC prevents UV-mediated EGFR phosphorylation at Y^992^ and Snail expression [70]. These studies suggest important roles for ROS and RNS in IR-induced activation of the EGFR pathway that may upregulate Snail to induce EMT and invasion. In addition, IR has been shown to induce Src activation [45, 106]. Src is a non-receptor tyrosine kinase that acts both upstream and downstream of EGFR and ErbB2. IR-induced Src activation promotes phosphorylation of EGFR and ErbB2 [45, 106]. Furthermore, IR-induced EGFR and IGFR-1 activation are known to promote the PI3K-dependent Rho signalling pathway, which enhances the invasive potential of glioblastoma cells [107].

IR has been shown to induce Akt activation through several signalling pathways (EGFR, C-X-C chemokine receptor type 4 [CXCR4]/C-X-C motif chemokine 12 [CXCL12], plasminogen activator inhibitor 1 [PAI-1]) and upstream regulators (Bmi1, PTEN) that promote EMT and invasion [81, 104, 109–111]. IR-mediated activation of EGFR leads to Akt activation through phosphorylation at two key regulatory residues, T308 and S473 [104]. ROS is also involved in IR-mediated Akt activation to enhance invasiveness. IR-induced ROS upregulates CXCR4, which interacts with its ligand, CXCL12, and activates the PI3K/Akt and ERK1/2 pathways [109].

PAI-1 signalling is also implicated in IR-induced Akt activation that increases Snail levels to induce EMT [81]. IR increases the expression and secretion of PAI-1 by upregulating HIF-1α, p53, and phospho-Smad3. PAI-1 secreted from radioresistant NSCLC cells induces EMT and the radioresistance of nearby cells in a paracrine manner; extracellular PAI-1 associates with the urokinase-type plasminogen activator (uPA)/uPAR complex and then binds to its receptor, low density LRP-1, which subsequently activates Akt and ERK1/2 to upregulate Snail, thereby inducing EMT and cell survival in radiosensitive cells [81]. IR also increases the expression of Bmi-1, which acts as an upstream regulator of the PI3K/Akt pathway. Bmi-1 is known as a key gene involved in EMT and the self-renewal of cancer cells [110]. In addition, IR downregulates PTEN to activate the PI3K/Akt pathway, which then inactivates GSK3β to increase Snail expression and induce EMT [111].

The IR-induced PI3K/Akt pathway also stabilises β-catenin, which directly binds to the promoter region of G-CSF. Subsequently, G-CSF is secreted and binds to G-CSFR to activate the JAK/STAT3 pathway [112]. STAT3 activation is also mediated by EGFR-Akt, as well as by the EGFR-p38/ERK pathway, in response to IR [113]. STAT3 is known to be involved in IR-induced EMT and invasion by upregulating the molecules governing EMT (N-cadherin, vimentin, uPA), invasion (MMP-2, MMP-9), and angiogenesis (vascular endothelial growth factor [VEGF], iNOS) [113–115]. In addition, IR-induced STAT3 also increases FoxM1 expression and it interacts and co-localizes with FoxM1 in the nucleus [117]. IR-induced FoxM1 directly binds to Snail promoter to induce Snail expression, thereby showing the involvement of STAT3/FoxM1 complex in EMT [92]. In addition, in radioresistant cervical cancer cells, IR induces K-Ras activation that promotes the c-Raf/p38 pathway to increase cell migration and metastatic potential [116].

### Induction of CSCs by IR

#### CSCs

CSCs possess a capacity for self-renewal, and they can persistently proliferate to initiate tumours upon serial transplantation, thus enabling them to maintain the whole tumour. Under certain microenvironment, CSCs exhibit plasticity; mutations in normal stem cells, progenitor cells, and/or differentiated cells can give rise to CSCs, and these newly generated CSCs produce daughter CSCs as well as differentiated bulk cancer cells [120–124]. Notably, some CSCs can spontaneously arise from normal and neoplastic nonstem cells, suggesting a bidirectional interconversion between the stem and non-stem cell state. Thus, different types of CSC coexist and contribute to tumour heterogeneity [120–123, 125]. Conventional cancer treatments kill most cancer cells, but CSCs survive due to their resistance to therapy, eventually leading to tumour relapse and metastasis [126–131].

For the identification of CSCs, three types of markers are utilised: cell surface molecules, transcription factors, and signalling pathway molecules [132–140]. CSCs express distinct and specific surface markers; commonly used ones are CD24, CD34, CD38, CD44, CD90, CD133, and ALDH. These markers enable CSCs to be distinguished from other tumour cells and from normal stem cells [132–140]. For example, breast CSCs express CD44^+^CD24^-^, while pancreatic or ovarian CSCs express CD44^+^CD24^+^EpCAM^+^ [135–137].

Transcription factors, including Oct4, Sox2, Nanog, c-Myc, and Klf4, and signalling pathways, including those of TGF-β, Wnt, Hedgehog, Notch, platelet-derived growth factor receptor (PDGFR), and JAK/STAT, are known to play crucial roles in maintaining the self-renewal abilities and pluripotency of stem cells [132–134]. These transcription factors and signalling pathways are also frequently used as CSC markers. In addition, several microRNAs (miRNAs), including let-7, miR-22, miR-34a, miR-128, the miR-200 family, and miR-451, are known to regulate the self-renewal, differentiation, and tumourigenicity of CSCs [141–143].

The CSC state can be regulated by cell-autonomous forces (genetic, epigenetic, and metabolic regulation) and by external forces (niche factors and the immune system) [120–123]. Non-CSCs can be reprogrammed to become CSCs by epigenetic and genetic changes that are involved in phenotypic heterogenicity among cancer cells [141–145]. Epigenetic changes, including DNA methylation, histone modifications, and miRNAs, play important roles in the acquisition of CSC properties.

In particular, miRNAs have been shown to play important roles in stemness and tumour metastasis; they modulate the expression of many target genes that regulate tumour cell EMT, motility, invasion, intravasation, resistance to anoikis, extravasation, and metastatic colonisation, as well as cell stemness, dormancy, metabolic reprogramming, and the TME. Through these means, miRNA can positively or negatively regulate tumour progression and tumour metastasis [141–143, 146–149]. In addition, long noncoding RNAs (lncRNAs) have been associated with numerous functions in cells [147, 150–154]. LncRNAs are known to positively or negatively affect the expression of nearby genes, control protein activity or localisation, and serve as organisational frameworks of subcellular structures. Many lncRNAs are also processed to yield small RNAs or to modulate other RNAs to be processed [154]. In particular, MALAT1, HOTAIR, and H19 lncRNAs are known to control stemness, cell migration and invasion, EMT, and metastasis by epigenetic regulation, alternative splicing, chromatin modification, and translational control [147, 150–153].

#### EMT and CSCs

EMT has been shown to play important roles in the acquisition of stemness in cancer cells [155–160]. EMT-inducing transcription factors, such as Snail, ZEB1, and Twist1, are known to confer CSC properties [161–165]. In addition to its role in EMT, Snail is known to induce the CSC phenotype in colorectal carcinoma cells, where it enhances stemness properties—including self-renewal, tumourigenicity, and resistance to radiotherapy/chemotherapy—with an increased metastatic potential [161–163].

ZEB1 is implicated in maintaining stemness and EMT properties in pancreatic and colorectal cancer cells [164]. ZEB1 represses the expression of stemness-inhibiting miRNAs, including miR-183, miR-200c, and miR-203, thereby upregulating the stem-cell factors Sox2 and Klf4. Knockdown of ZEB1 prevents not only EMT, invasion, and metastasis, but also the stemness phenotype [164]. In addition, Twist1 is known to link EMT to stem-like features. Twist1 directly increases Bmi-1 expression, and acts cooperatively with Bmi-1 to induce EMT and stemness properties [165].

Signalling pathways involved in EMT, including those of TGF-β, Wnt, and Notch, have been shown to play important roles in inducing the CSC phenotype [166–168]. TGF-β1 not only increases EMT markers (Slug, Twist1, β-catenin, N-cadherin), but also upregulates CSC markers (Oct4, Sox2, Nanog, Klf4) in breast and lung cancer cells [166, 167].

Wnt/β-catenin signalling also plays critical roles in increasing the stemness properties of liver CSCs by activating Notch1 [168]. Blocking Wnt/β-catenin and/or Notch decreases the expression of transcription factors involving EMT (such as Snail) and stemness (such as Sox2 and Nanog). These changes result in reduced metastatic potential in vivo, and they inhibit CSC properties, including self-renewal and tumourigenicity. This suggests a role for EMT in the acquisition of CSC phenotypes [168].

However, in heterogeneous solid tumours, some CSC subpopulations arise independently of EMT [169, 170]. This suggests that CSC populations may be heterogeneous, and may contain a significant proportion of epithelial stem cells in which stemness is entirely uncoupled from EMT. These epithelial stem cells may cooperatively interact with non-CSCs, thereby potentiating the metastatic behaviours of the combined tumour cell populations [171–174]. Therefore, other mechanisms are likely involved in the induction of CSC in an EMT transcription factors-independent manner.

#### Induction of the CSC phenotype by IR

IR has been shown to induce the CSC phenotype in many cancers, including breast, lung, and prostate cancers, as well as melanoma [175–181]. Genotoxic stress due to IR or chemotherapy promotes a CSC-like phenotype by increasing ROS production [179]. IR has been shown to induce reprogramming of differentiated cancer cells into CSCs [181]. In prostate cancer patients, radiotherapy increases the CD44^+^ cell population that exhibit CSC properties [175]. IR also induces the re-expression of stem cell regulators, such as Sox2, Oct4, Nanog, and Klf4, to promote stemness in cancer cells [176, 181].

EMT has been implicated in the acquisition of the IR-induced CSC phenotype [178, 179]. After IR, surviving cells exhibit a complex phenotype combining the properties of EMT and CSC with high expression levels of Snail, CD24, CD44, and PDGFR-β in NSCLC cells [178]. In addition, the subset of CD24^+^ ovarian cancer cells or CD133^+^ colorectal cancer cells that possess CSC properties exhibit the EMT phenotype—including higher levels of expression of Snail, Twist, and vimentin, and lower levels of expression of E-cadherin [159, 160].

EMT-inducing transcription factors and signalling pathways, including Snail, STAT3, Notch signalling, the PI3K/Akt pathway, and the MAPK cascade, have been shown to play important roles in IR-induced CSC properties [180–184]. STAT3 has been shown to be involved in the IR-induced increase of CSCs [180], and is known to activate Snail to induce the CSC phenotype. STAT3 directly binds to the Snail promoter and increases Snail transcription, which induces the EMT and CSC phenotypes, in cisplatin-selected resistant cells [163]. Inhibition of the DNA-binding activity of STAT3 prevents IR-induced increases of the CSC population, and sensitises cells to radiotherapy [180].

Notch signalling is also implicated in the IR-induced *de novo* generation of CSCs [181, 184]. Inhibition of Notch signalling partially prevents the IR-induced re-expression of Oct4, Sox2, Nanog, and Klf4 [181]. Notch signalling also plays important roles in the IR-induced metastatic potential of CSCs. IR upregulates disintegrin and metalloproteinase-17 (ADAM17) to activate Notch signalling, which increases the migration and invasiveness of CSCs [182].

The PI3K/Akt pathway and the MAPK cascade are involved in the IR-induced CSC and EMT phenotypes. IR promotes Src activity to trigger the PI3K/AKT and p38 MAPK pathways that induce both CSC status and EMT [183]. Therefore, EMT transcription factors and signalling pathways may enable CSCs to acquire the ability to invade, migrate, and disseminate.

### Induction of oncogenic metabolism by IR

#### Oncogenic metabolism

Most cancer cells produce their energy predominantly by high rate of glycolysis rather than by oxidative phosphorylation, even in the presence of oxygen: a phenomenon that has been termed the Warburg effect, aerobic glycolysis, or the glycolytic switch [185–194]. Other oncogenic metabolic pathways, including glutamine metabolism, the pentose phosphate pathway (PPP), and synthesis of fatty acids and cholesterol, are also enhanced in many cancers. These alterations are known to contribute to cell survival and sustain the increased demands of cell proliferation by providing biosynthetic precursors for nucleic acids, lipids, and proteins [186–196].

The activation of oncogenes and the loss of tumour suppressors have been shown to drive tumour progression; in particular, they seem to drive metabolic reprogramming. Several transcription factors, including HIF-1α, p53, and c-Myc, are known to contribute to oncogenic metabolism [186–194]. Emerging evidence suggests that metabolic reprogramming is one of the hallmarks of cancer, and may be required to convert a normal cell into a malignant cell [186–194].

Although the Warburg effect has been considered a metabolic signature of tumour cells, increasing evidence indicates that tumour cells exhibit high mitochondrial metabolism as well as aerobic glycolysis. These contradictory findings have even been reported as occurring within the same tumour [197–208]. In addition, CSCs exhibit unique metabolic features in a tumour type-dependent manner. CSCs can be highly glycolytic-dependent or oxidative phosphorylation (OXPHOS)-dependent. In any case, mitochondrial function is crucial for maintaining CSC functionality [209–212]. To explain such contradiction, reverse Warburg effects and metabolic symbiosis have been proposed [197–208, 212].

According to this model, cancer cells depend on mitochondrial metabolism and increase mitochondrial production of ROS that cause pseudo-hypoxia. Tumour tissue is a heterogeneous population of cells consisting of cancer cells and surrounding stromal cells, with various genetic and epigenetic backgrounds. These ROS reduce caveolin-1 expression in cancer-associated fibroblasts (CAFs), which are the main component of tumour stroma. Loss of caveolin-1 in CAFs leads to further increases in ROS production, which stabilise HIF-1α (and by extension, this increases levels of the HIF-1 heterodimer). HIF-1 then enhances glycolysis in CAFs. Furthermore, tumour cell-derived ROS also induce autophagy in CAFs. Autophagy is a lysosomal self-degradation process that removes damaged mitochondria through mitophagy. Thus, CAFs have defective mitochondria that lead to the cells exhibiting the Warburg effect; the cells take up glucose, and then secrete lactate to 'feed' adjacent cancer cells [197–207].

In tumour tissue, epithelial cancer cells and CAFs express different subtypes of the lactate transporter, monocarboxylate transporter (MCT). This heterogeneity of MCT expression induces metabolic symbiosis between epithelial cancer cells and CAFs. Metabolic symbiosis is required for adaptation to changes in the nutrient microenvironment that is caused by cancer treatment. Epithelial cancer cells express MCT1, while CAFs express MCT4. MCT4-positive, hypoxic CAFs secrete lactate by aerobic glycolysis, and MCT1-expressing epithelial cancer cells then uptake and use that lactate as a substrate for the tricarboxylic acid (TCA) cycle [197–201].

However, the reverse Warburg effect may not be pervasive in all cancers. MCT4-expressing tumour cells or the mesenchymal phenotype do not lead to the reverse Warburg phenomenon. Rather, hierarchical metabolic heterogeneity may be observed in cancer cells; MCT4-positive cancer cells depend on glycolysis and then efflux lactate, while MCT1-positive cells uptake lactate and rely on OXPHOS. Therefore, metabolic heterogeneity induces a lactate shuttle between hypoxic/glycolytic cells and oxidative/aerobic tumour cells. This kind of lactate shuttle has also been observed between neurons and astrocytes in normal brain tissue [198, 200].

This interaction between cancer cells and stromal cells can contribute to tumour progression—including tumour EMT, invasion, growth, and angiogenesis. Cancer cells interact with stromal cells and use their environment to sustain tumour growth. In addition, cells in the tissues surrounding the tumour, such as CAFs and adipocytes, create a nutrient-rich microenvironment that feeds the cancer cells; cancer cells then secrete waste products (e.g., CO_2_, H^+^, ammonia, polyamines) that further promote EMT, invasion, and angiogenesis [198, 200, 208].

MCT1-positive cancer cells are also involved in the stem-like phenotypes observed within heterogeneous tumour populations. While bulk tumour cells exhibit a glycolytic phenotype, with increased conversion of glucose to lactate (and enhanced lactate efflux through MCT4), CSC subsets depend on oxidative phosphorylation; most of the glucose entering the cells is converted to pyruvate to fuel the TCA cycle and the electron transport chain (ETC), thereby increasing mitochondrial ROS production [198, 209, 212]. In these cells, the major fraction of glucose is directed into the pentose phosphate pathway, to produce redox power through the generation of NADPH and ROS scavengers [212]. Therefore, this activated mitochondrial metabolism provides enough energy for CSC self-renewal, invasion, and metastasis.

#### EMT/CSC regulators involved in oncogenic metabolism

Several transcription factors, including HIF-1α, p53, and c-Myc, are known to contribute to oncogenic metabolism. Many regulatory molecules involved in EMT and CSCs, including Snail, Dlx-2, HIF-1, STAT3, TGF-β, Wnt, and Akt, are implicated in the metabolic reprogramming of cancer cells. The induction of EMT is involved in the acquisition of CSC properties, as well as in reduced mitochondrial metabolism and induction of the glycolytic switch [57, 58, 213–222].

Snail has been shown to induce mitochondrial repression and glucose metabolism by downregulating cytochrome C oxidase (COX) subunits or fructose-1,6-bisphosphatase 1 (FBP1). Snail has also been shown to induce the EMT phenotype [57, 58, 213–215].

HIF-1 induces the expression of glycolytic enzymes, including the glucose transporter GLUT, hexokinase, lactate dehydrogenase (LDH), and MCT, resulting in the glycolytic switch. In addition, HIF-1 represses the expression of pyruvate dehydrogenase kinase (PDK), which inhibits pyruvate dehydrogenase (PDH), thereby inhibiting mitochondrial activity [216, 217].

STAT3 has been implicated in EMT-induced metabolic changes as well [218]. Stable EMT cells are generated through mammosphere culture in epithelial breast cancer cells. These EMT-derived cancer cells exhibit elevated activation of STAT3 and enhanced aerobic glycolysis, with upregulation of certain enzymes and transporters related to glycolysis (such as MCT2); these cells also show downregulation of gluconeogenesis and some anabolic side-pathways. Inhibition of STAT3 suppresses certain EMT-related metabolic alterations in the expression of MCT2 and ZEB1, suggesting a role for STAT3 in EMT-induced metabolic changes [218].

Emerging evidence suggests that TGF-β and Wnt play important roles in the metabolic alteration of cancer cells [57, 58, 214, 219–221]. TGF-β and Wnt are known to induce mitochondrial repression and the glycolytic switch by activating Dlx-2 and Snail [57, 58]. TGF-β/Wnt-induced mitochondrial repression is mediated by inhibition of mitochondrial complex IV (COX) [57, 214]. Wnt also directly targets PDK1, thereby inhibiting mitochondrial respiration and promoting the glycolytic switch [219, 221].

Akt is also implicated in the glycolytic switch and in promoting cancer cell invasiveness [222]. Overexpression of Akt impairs mitochondrial function, promotes glycolytic metabolism with upregulation of glyceraldehyde-3-phosphate dehydrogenase (GAPDH), and converts radial growth (i.e., noninvasive) melanoma into vertical growth (i.e., invasive) melanoma [222].

#### Oncogenic metabolism plays a critical role(s) in EMT and CSC phenotypes

Accumulating evidence suggests that metabolic alteration is one of the hallmarks of cancer, and may contribute to malignant transformation and tumour development—including the induction of EMT, invasion, metastasis, and stemness [58, 211–213, 223–233] (Fig. 1). Metabolic reprogramming of cells toward aerobic glycolysis has been shown to support the invasive phenotype of malignant melanoma [224]. A glycolytic mechanism is also known to modulate the angiogenic switch for metastatic growth [225].

Several glycolytic enzymes, including pyruvate kinase M2 (PKM2), LDH, and pyruvate carboxylase (PC), are implicated in the induction of the EMT and CSC phenotypes [234–237]. PKM2 is a less active isoform of pyruvate kinase and is primarily expressed in embryonic and cancer cells. This decreased activity of PKM2 is known to promote an overall shift in metabolism to aerobic glycolysis. EMT-inducing stimuli cause nuclear translocation of PKM2, which promotes EMT; nuclear PKM2 directly interacts with TGF-β-induced factor homeobox 2 (TGIF2), a transcriptional repressor of TGF-β signalling, and recruits histone deacetylase 3 to the E-cadherin promoter to suppress E-cadherin transcription [234].

LDH catalyses the bidirectional conversion of lactate to pyruvate [237]. LDHA is one of the predominant isoforms of LDH; it is also known to be implicated in the Warburg effect, as well as in cell invasion and migration. High levels of LDHA are positively correlated with the expression of EMT and CSC markers in invasive bladder cell lines and in muscle-invasive bladder cancer specimens, suggesting a critical role for LDHA in the activation of EMT and CSC [237].

In addition, PC is implicated in cell migration and invasion [236]. PC is a key enzyme of anaplerosis that converts pyruvate to oxaloacetate, which replenishes the TCA cycle. Knockdown of PC inhibits proliferation, migration, and invasion behaviours in invasive breast cancer cells; conversely, the overexpression of PC promotes proliferation, migration, and invasion abilities in noninvasive breast cancer cells [236].

Furthermore, the misregulation of lipogenic metabolism is involved in the regulation of EMT [238, 239]. Fatty acid synthase (FASN) is a key lipogenic enzyme that catalyses *de novo* synthesis of fatty acids. FASN signalling is known to modulate subcellular structural components that determine the epithelial or mesenchymal state of a cell. Transient knockdown of FASN suppresses structural hallmarks of EMT in stem-like cells. Loss of FASN signalling also reverses a tumour phenotype to a normal-like tissue phenotype, and efficiently suppresses the tumourigenicity of metastatic breast cancer cells in vivo [238]. Mechastically, FASN increases TGF-β levels and TGF-β, in turn, elevates FASN expression. These results suggest that a FASN-TGF-β-FASN positive loop contributes to high EMT/metastatic potential in cisplatin resistant cancer cells [239].

Interestingly, the respiratory enzymes citrate synthase (CS) and succinate dehydrogenase subunit B (SDHB), and the gluconeogenesis regulatory enzyme FBP, are known to negatively regulate the EMT and CSC phenotypes [215, 240, 241]. Loss of CS has been shown to induce EMT and the glycolytic switch. CS is a mitochondrial respiratory enzyme that catalyses the first step of the TCA cycle. CS knockdown cells exhibit EMT, mitochondrial repression, and the glycolytic switch, with concomitant upregulation of Snail and Twist, and downregulation of p53 and its target genes (TIGAR and SCO2). p53 is known to prevent glycolysis and promote mitochondrial respiration by increasing the expression of TIGAR and SCO2. p53 reactivation inhibits CS-knockdown-induced EMT, suggesting a role for p53 in these metabolic alterations and in malignant transformation [240].

SDHB is also implicated in EMT, glucose and glutamine metabolism, and mitochondrial dysfunction. SDH is a mitochondrial metabolic enzyme complex that participates in both the TCA cycle and the electron transport chain; it converts succinate into fumarate in the TCA cycle and catalyses the transfer of electrons to the ubiquinone pool in the electron transport chain. SDH mutations have frequently been observed in many cancers. Knockdown of SDHB leads to alterations of the epigenome; this promotes EMT, induces altered glucose and glutamine utilisation, and induces mitochondrial dysfunction [241].

In addition, loss of FBP has been associated with the EMT-driven CSC phenotype. FBP catalyses the conversion of fructose 1,6-bisphosphate to fructose-6-phosphate. Snail induces epigenetic silencing of FBP1; this enhances glycolysis, suppresses oxygen consumption and ROS production, and promotes the EMT and CSC phenotypes [215].

We also showed that glutamine metabolism plays an important role in the induction of EMT [58]. Glutaminase 1 (GLS1) converts glutamine to glutamate. The inhibition of glutamine metabolism (via GLS1 knockdown, glutamine deprivation, or glutamine metabolism inhibitors) suppressed Dlx-2-, TGF-β-, Wnt-, and Snail-induced EMT and the glycolytic switch. In addition, GLS1 knockdown also suppressed tumour growth and metastasis in vivo. Dlx-2 knockdown and glutamine metabolism inhibition decreased Snail mRNA levels through the p53-dependent upregulation of Snail-targeting microRNAs (miR-23b, miR-29b, miR-30, miR-34, miR-125b, miR-148a, miR-153, miR-200, and miR-203). These results indicate that the Dlx-2/GLS1/glutamine metabolic axis is a crucial regulator of TGF-β/Wnt-induced, Snail-dependent EMT, metastasis, and the glycolytic switch [58].

Oncogenic metabolism, including glutamine metabolism, is known to endow cancer cells with growth advantages by providing biosynthetic precursors [187–196]. Given that GLS1 knockdown suppressed tumour growth and metastasis in vivo, it is possible that knockdown of any component enzyme in oncogenic metabolism results in a pronounced suppression of metastasis. Like GLS1, other enzymes in oncogenic metabolism may also regulate p53-dependent modulation of Snail-targeting microRNAs to mediate Snail-induced EMT. Therefore, we propose that all oncogenic metabolic pathways are interconnected so that inhibition of any component enzyme within the overall oncogenic metabolism may suppress EMT. Further studies are needed to determine which enzyme inhibition is the most effective in producing EMT inhibition.

#### IR induces oncogenic metabolism

IR has been shown to induce metabolic changes in cancer cells [242–247]. IR enhances glycolysis by upregulating GAPDH (a glycolysis enzyme), and it increases lactate production by activating LDHA, which converts pyruvate to lactate. IR also elevates MCT1 expression that exports lactate into the extracellular environment, leading to acidification of the tumour microenvironment. These changes are associated with IR-induced invasion of the non-irradiated, surrounding breast cancer tissues and normal endothelial cells [243].

IR increases intracellular glucose, glucose 6-phosphate, fructose, and products of pyruvate (lactate and alanine), suggesting a role for IR in the upregulation of cytosolic aerobic glycolysis; this was also revealed in the metabolomic profile of hepatoma cells [246]. Lactate can activate latent TGF-β through a pH-dependent mechanism so that LDHA inhibition prevents radiation-induced activation of TGF-β [247]. In addition, lactate stimulates cell migration and enhances secretion of hyaluronan from CAF that promote tumour metastasis [235]. In addition to glycolysis, IR has been shown to affect other components of oncogenic metabolism. For example, radioresistant head and neck squamous cells exhibit profound alterations in their metabolism; they demonstrate increased glucose uptake, enhanced PPP signalling, and increased fatty acid biosynthesis, while also showing decreased mitochondrial oxidative phosphorylation [245].

ROS are known to play important roles in the IR-induced glycolytic switch [242]. IR-induced ROS generation increases tumour glucose uptake in vivo. An antioxidant SOD mimic prevents IR-induced glucose uptake, forestalls the glycolytic switch, and inhibits invasiveness [242]. IR-induced ROS generation is known to increase the activity of transcription factors and inducers that are involved in the EMT and CSC phenotypes, such as Snail, Dlx-2, HIF-1, and TGF-β. These factors have been shown to regulate the enzymes involved in glycolysis and mitochondrial oxidative phosphorylation, which may be involved in the IR-induced glycolytic switch.

Snail has been shown to induce the glycolytic switch with EMT phenotypes [57, 58, 213–215]. Because Snail is known to be induced by IR [53–56], we investigated whether Snail affected the IR-induced glycolytic switch (data not shown). We found that IR increases glucose consumption and lactate production, and decreases O_2_ consumption; this indicates that IR induces mitochondrial repression and the glycolytic switch in MCF-7 cells. Conversely, Snail shRNA prevented IR-induced mitochondrial repression and glycolytic switch, indicating that IR induces these phenomena via Snail.

Dlx-2 shRNA also decreased the IR-induced glycolytic switch and mitochondrial repression, and resulted in the downregulation of Snail. Thus, the Dlx-2/Snail axis seems to be implicated in the IR-induced glycolytic switch. Using cDNA microarray technology, we also found that Dlx-2 elevates a key enzyme in glutamine metabolism, GLS1, and that the Dlx-2/GLS1/Gln metabolic axis plays important roles in TGF-β/Wnt/Snail-dependent EMT and in the glycolytic switch [58]. These results suggest that Dlx-2 may be implicated in IR-induced alterations of other oncogenic metabolic pathways. In addition, we found that GLS1 knockdown inhibits IR-induced EMT (data not shown).

HIF-1 is also implicated in IR-induced metabolic alterations [244]. IR increases HIF-1α expression that inhibits PDH and the tricarboxylic acid cycle, and triggers a metabolic switch to increase lactate production [244].

As described above, metabolic changes have been implicated as being closely involved in the acquisition of the EMT and CSC phenotypes [58, 211–213, 223–233]. IR may indirectly activate several signalling pathways through ROS production, and may induce the activation of oncogenes or the inactivation of tumour suppressors, which then leads to metabolic alterations, EMT, and stemness phenotypes. Therefore, IR appears to induce the EMT and CSC phenotypes by promoting oncogenic metabolism.

Similarly, UV radiation is known to induce the Warburg effect to promote melanoma invasion. UV radiation increases glucose consumption and lactate production, which is partly mediated by ROS. Lactic acid then enhances the invasive potential of melanoma cells. UV radiation also upregulates Transketolase (an enzyme of the PPP) and activates Akt, both of which are involved in metabolic changes [248].

### Changes in TME by IR

Crosstalk between cancer cells and their microenvironment is critical for invasive growth and metastasis. The TME is composed of ECM and multiple cell types, including fibroblasts, vascular endothelial cells, immune cells, pericytes, and adipocytes. Cancer cells secrete multiple factors, such as growth factors, cytokines, and chemokines, that regulate the phenotype and function of tumour-resident cells and that influence the composition and organisation of the ECM, thereby regulating such qualities as tumour stiffness [36, 249–253]. IR can elicit various changes in the TME. These changes contribute to creating a favourable microenvironment for tumour metastasis and for the self-renewal and maintenance of cancer stem cells [87, 249–253].

### TME

1. Cancer-associated fibroblasts (CAFs)
  Fibroblasts are derived from mesenchyme; they form the structural framework in tissues, and typically prevent tumour formation. Unlike normal fibroblasts, CAFs do the following: promote tumour survival, growth, invasion, and metastasis; enhance the stiffness of the ECM; contribute to angiogenesis; and induce inflammation by releasing several growth factors and cytokines (TGF-β, VEGF, hepatocyte growth factor [HGF], PDGF, and stromal cell-derived factor 1 [SDF1]), as well as MMP [249, 254–256]. Recent studies have demonstrated that CAFs also exert tumour-suppressive effects through direct suppression of cancer cells and via regulation of immune cell behaviour. Although some debate exists on this subject, CAFs are predominantly assigned a tumour-promoting function [254].

2. Vascular endothelial cells
  The tumour vascular network is dynamic and is associated with tumour growth. A growing tumour requires a constant supply of oxygen, nutrients, and blood-borne mitogens, and requires an effective way to remove toxic metabolites. Thus, tumours recruit the host tissue’s blood vessel network to perform four mechanisms: angiogenesis (formation of new vessels), vasculogenesis (*de novo* formation of blood vessels from endothelial precursor cells), co-option, and modification of existing vessels within tissues. These mechanisms are required for continuous tumour growth and metastatic potential [36, 249, 252].

3. Immune cells
  The immune infiltrate can be composed of a variety of different cell types. These cell populations can have both pro- and anti-tumour functions, and can vary in their activation status and their localisation within the tumour. Innate (macrophages, dendritic cells, myeloid-derived suppressor cells (MDSCs), natural killer cells, etc.) and adaptive (T and B cells) immune system components play major roles in the regulation of tumour growth [257, 258]. Although immune cells have commonly been accepted to exert anti-tumour responses, mechanisms of immune suppression can prevent this process. These immune suppression networks include the immunosuppressive cells such as tumour-associated macrophages (TAM), MDSCs, and regulatory T cells, and the immunosuppressive cytokines, TGF-β and interleukin-10 (IL-10) [259]. Cancer cells interact with the immune system, and can either reduce its intrinsic immunogenicity or induce tolerance [249, 260, 261].
  This tumour-host immune relationship is referred to as ‘cancer immunoediting’, which is described by three phases: 1) elimination, 2) equilibrium, and 3) escape. In the elimination phase, highly immunogenic transformed cells are immediately recognised and destroyed by both the innate and adaptive immune systems. In the equilibrium phase, some tumours elude the initial host defences and coexist with the adaptive immune system. In this phase, tumours try to grow but they are inhibited by the immune system. The third phase, tumour escape, is mediated by antigen loss, immunosuppressive cells (TAM, MDSCs, and regulatory T cells), and immunosuppressive cytokines (TGF-β and IL-10). Various types of immunotherapy try to shift the tumour from the escape phase and equilibrium phase to the elimination phase [36, 261]. Heterogeneity in the tumour immune system is associated with various factors, including CAF-secreted factors, vasculature permeability, and the tumour cells themselves [249].

#### Changes in TME by IR

IR can elicit various changes in the TME, such as CAF activity-mediated ECM remodelling and fibrosis, cycling hypoxia, and an inflammatory response [87, 249–253] (Fig. 3). IR activates CAFs to promote the release of growth factors and ECM modulators, including TGF-β and MMP. TGF-β is a major CAF-secreted factor [87, 255, 256]. TGF-β directly influences tumour cells and CAFs, promotes tumour immune escape, and activates HIF-1 signalling [87, 252, 255]. MMPs degrade ECM that facilitates angiogenesis, tumour cell invasion, and metastasis [262]. IR also promotes MMP-2/9 activation in cancer cells to promote EMT, invasion, and metastasis [54, 106, 263–266]. IR enhances MMP-2 transcription and protein secretion by activating the EGFR/p38/Akt and EGFR/PI3K/Akt signalling pathways, which enhance the invasion of glioma cells [106]. IR-induced Snail increases MMP-2 expression to promote EMT [54]. IR also increases MMP-9 expression by activating the PI3K/Akt/NF-κB pathway, which enhances hepatocellular carcinoma cell invasion [263]. IR-induced MMP-2/MMP-9 expression not only degrades ECM proteins, but also cleaves latent TGF-β1 to activate the TME [266].

**Fig. 3:** IR-induced side effects on cancer cells and the tumour microenvironment (TME). Radiotherapy has the paradoxical side-effect of increasing tumour aggressiveness. IR promotes ROS production in cancer cells, which may induce the activation of oncogenes and the inactivation of tumour suppressors, which further promote oncogenic metabolism. Metabolic alterations are involved in tumour progression, and include growth, invasion, metastasis, and the acquisition of the CSC phenotype, thereby contributing to tumour recurrence and distant metastasis. Given that IR induces EMT and CSC properties in cancer cells, it is possible that IR-induced oncogenic metabolism is required for the acquisition of the EMT and CSC phenotypes. IR can also elicit various changes in the TME, such as: 1) the emergence of cancer-associated fibroblasts (CAFs), activity-mediated extracellular matrix (ECM) remodelling, and fibrosis, 2) cycling hypoxia, and 3) an inflammatory response. IR activates cancer-associated fibroblasts (CAFs) to promote the release of growth factors, including transforming growth factor-β (TGF-β), and extracellular matrix (ECM) modulators, including matrix metalloproteinase (MMP). TGF-β directly affects tumour cells and CAFs, enhances tumour immune escape, and activates hypoxia-inducible factor-1 (HIF-1) signalling. MMPs degrade the ECM, facilitating tumour invasion and metastasis. IR can also cause damage to the vascular endothelial cells (EC), leading to hypoxia that further promotes HIF-1 signalling. HIF-1 increases the expression of vascular endothelial growth factor (VEGF) and chemokine (C-X-C motif) ligand 12 (CXCL12), both of which induce angiogenesis and vasculogenesis. IR also upregulates integrins on ECs that enhance survival and confer radioresistance. Although IR activates an antitumour immune response, this signalling is frequently suppressed by tumour escape mechanisms (such as programmed cell death protein 1 ligand 1 [PDL1] signalling) and by suppressive immune cells (regulatory T cells [Treg], myeloid-derived suppressor cells [MDSC], and tumour-associated macrophages [TAM]), which are relatively less radiosensitive than other lymphocyte subsets. These IR-mediated changes in the TME may constitute additional adverse effects of IR on the patient by promoting angiogenesis, invasion, metastasis, and radioresistance

IR can also damage endothelial cells, resulting in hypoxia that further promotes HIF-1 signalling. HIF-1 induces angiogenesis and vasculogenesis through the upregulation of VEGF and CXCL12 [75, 267–271]. VEGF is known to be induced by various upstream activators, such as environmental cues, growth factors, cytokines, hormones, and oncogenes. IR increases VEGF expression by upregulating HIF-1α and NF-κB in prostate cancer [269, 270]. As mentioned above, IR also induces the reoxygenation of hypoxic cancer cells to activate HIF-1 signalling. IR-induced reoxygenation also enhances the translation and secretion of HIF-1-regulated genes and VEGF, thereby increasing endothelial cell radioresistance [77]. Inhibition of HIF-1α/VEGF-A signalling enhances radiosensitivity [271]. Notably, the hypoxic regions of tumours can function as a refuge for CSCs, and increase their survival during chemotherapy. In addition, stem cell-like properties could be induced by paracrine signalling from endothelial cells, thereby increasing chemoresistance [249]. Furthermore, IR also upregulates integrins on endothelial cells, which enhances their survival and confers radioresistance [249, 252].

Endothelial cell damage also leads to initiation of inflammatory signalling and increased attraction of innate immune cells [75, 267, 268]. Although IR stimulates an immune response by inducing damage-associated molecular pattern (DAMP) and NKG2D signalling in cancer cells, this signalling is frequently suppressed by regulatory T cells, which leads to immune tolerance. Other tumour escape mechanisms, such as programmed cell death protein 1 ligand 1 (PDL1) signalling and MDSC/TAM-derived IL-10 immunosuppression, also remain intact. In addition, after radiotherapy, the number of these locally immunosuppressive cells (TAM, MDSCs, and regulatory T cells) is relatively high owing to their lower radiosensitivity compared to other lymphocyte subsets [252, 260, 261].

These IR-mediated changes in the TME may be additional adverse effects of IR by promoting radioresistance, tumour recurrence, and metastasis. The roles of the TME in determining radiotherapy outcomes have been reviewed elsewhere, and are not discussed in detail here.

### The roles of EMT, CSC, and oncogenic metabolism in radioresistance

More than half of cancer patients receive radiotherapy, with varying success. The dose of IR delivered to the tumour is limited by the risk of damage to the surrounding normal tissues. Therefore, radiation therapy aims to minimise the toxicity to normal tissues in the first approach, while maximising doses to cancer cells in the second approach. Three main biological factors of tumours can influence treatment outcome: 1) the intrinsic radioresistance of the cancer cells, 2) the repopulation capacity of surviving cancer cells during the intervals between treatments, and 3) the degree of hypoxia in the tissue environment [4, 272].

Radioresistance has been shown to arise from the activation of several different pathways, including survival pathways (PI3K/Akt, ERK), DNA DSB repair pathways (homologous recombination and non-homologous end-joining [NHEJ]), glycolysis, and autophagy. Radioresistance has also been shown to arise from the induction of cell cycle redistribution, and the inactivation of the apoptosis pathway, that follows exposure to radiation [272–275]. EMT, CSCs, and oncogenic metabolism play important roles in the development of cancer radioresistance by activating these pathways. Understanding these mechanisms is important to be able to develop new strategies to enhance cancer radiotherapy.

#### The roles of EMT signalling pathways in radioresistance

EMT has been shown to confer resistance to radiation and chemotherapy in many cancers [273–277]. After IR, surviving cells exhibit an EMT phenotype with upregulation of EMT markers, including Snail, Slug, ZEB1, Twist1, vimentin, and N-cadherin, in lung adenocarcinoma cells [277]. Cells undergoing EMT also exhibit increased radioresistance by acquiring stem-like properties, preventing apoptosis, enhancing survival pathways, and activating signalling pathways involved in cell cycle progression and DNA damage repair [273–275].

EMT-promoting transcription factors, including Snail, Slug, ZEB1, and ZEB2, are known to be associated with radioresistance [43, 278–286]. Snail is known to play important roles in radioresistance by inhibiting p53-mediated apoptosis, activating survival pathways, and inducing stem cell properties [278, 279]. IR induces apoptosis by upregulating the p53 target gene PTEN, a negative regulator of the PI3K/Akt survival pathway. Snail protein is stabilised by IR and subsequently binds to the PTEN promoter that inhibit p53 binding to the PTEN promoter. Thus, Snail prevents IR-mediated PTEN upregulation and activates the Akt pathway, thereby increasing radioresistance [278].

Slug is also known to be involved in radioresistance by inhibiting p53-mediated apoptosis and activating stem cell properties [279–282]. Slug knockout mice exhibited increased radiosensitivity [280, 281]. IR upregulates Slug by activating p53; Slug then directly represses p53-target gene PUMA transcription, thereby preventing IR-induced apoptosis [281]. Slug also induces CSC activity and radioresistance [279, 282]. Long non-coding RNA MALAT1 regulates Slug expression by reciprocally repressing miR-1, which contributes to CSC activity and radioresistance [282]. IR-induced Snail and Slug also promote EMT and stem cell properties, and they suppress p53-mediated apoptosis [279]. All these events help cancer cells to escape to newer and less adverse niches, generate the critical tumour mass necessary to form macrometastases, and survive under stress conditions in the primary tumour [279].

In addition, ZEB1 and ZEB2 have been associated with radioresistance [283–286]. ZEB1 is known to confer radioresistance by activating DNA damage repair pathways [283]. IR-induced DNA damage increases ATM activation that stabilises ZEB1. ZEB1, in turn, directly binds to USP7 deubiquitinase to stabilise CHK1, thereby activating the recombination-dependent DNA repair response. ZEB1 inhibition enhances radiosensitivity, but has no effect on EMT [283]. Consistent with this observation, ZEB2 also protects cancer cells from IR-induced apoptosis by inhibiting ATM/ATR activation in an EMT-independent manner [285]. These observations suggest EMT-independent roles for these transcription factors in radioresistance, but contradictory evidence also exists: ZEB1-induced EMT is involved in the radioresistance of nasopharyngeal carcinoma cells [284]. Therefore, further studies are needed to precisely determine the contribution of EMT and EMT-inducing transcription factors in responses to cancer therapy.

The signalling pathways involved in EMT, including those of TGF-β, Wnt, Notch, Hedgehog, and EGFR, are also known to be involved in radioresistance [90, 287–302]. TGF-β has been shown to play critical roles in radioresistance by inducing CSC properties and by activating DNA repair pathways [287–291]. TGF-β is known to promote IR-induced self-renewal pathways, including Notch1, and to induce effective DNA damage responses that lead to the radioresistance of glioblastoma-initiating cells [288]. TGF-β activates the NHEJ DNA repair pathway upon IR, by upregulating LIG4 (a DNA ligase in DNA DSB repair), thereby protecting cells from IR [290].

It is generally agreed that TGF-β switches from a tumour suppressor (in an early stage of tumourigenesis) to a tumour promoter (in a later stage of tumourigenesis) [37, 38]. Thus, the role of the TGF-β pathway in radiotherapy is still a matter of debate. However, inhibition of TGF-β signalling has been shown to increase radiosensitivity in vitro and enhance IR-induced tumour growth delay in vivo [287]. Inhibition of TGF-β also prevents IR-induced metastases in tumour-bearing mice [90]. In addition, increased circulating TGF-β levels during radiotherapy have been strongly correlated with poor prognoses for patients with non-small cell lung cancer [291].

Wnt/β-catenin signalling has been shown to confer radioresistance by enhancing stemness, by activating survival pathways, and by activating DNA damage repair pathways [292–296]. High Wnt signalling activity is associated with increased stemness and radioresistance in colorectal cancer cells and intestinal stem cells [296]. IR selectively increases β-catenin expression and nuclear localisation in progenitor cells, but not in nonprogenitor cells. β-catenin then enhances cell survival, partly by upregulating survivin, an apoptosis inhibitor [292, 293]. β-catenin also promotes the self-renewal of progenitor cells [293]. These behaviours may lead to increases in the IR-induced enrichment of progenitor cells, and may further enhance their radioresistance [292]. In addition, β-catenin activates the NHEJ DNA repair pathway by directly promoting LIG4 transcription, thereby increasing radioresistance [296]. Supporting this observation, nuclear β-catenin expression has been highly correlated with poor outcomes after radiotherapy in patients with cervical squamous cell carcinoma [294].

In addition, Notch signalling is associated with radioresistance by preventing apoptosis and enhancing survival pathways. Notch signalling confers radioresistance to glioma cells by activating the PI3K/Akt pathway and increasing expression of Mcl-1, an anti-apoptotic Bcl-2 family protein [297]. Akt activation is also mediated by EGFR signalling, and also increases radioresistance [298]. The PI3K/Akt/mTOR pathway promotes the EMT and CSC phenotypes via elevated levels of Snail, thereby increasing radioresistance [299]. Increased Akt Ser (473) phosphorylation and mTORC1 protein expression are also associated with enhanced EMT and radioresistance [301].

Furthermore, Hedgehog signalling is involved in radioresistance [302]. GLI1 proteins are the transcription factors of the Hedgehog effector. IR triggers the mTOR/S6K1 pathway that increases expression and nuclear translocation of GLI1, accompanied by increased expression of Snail. These events and components mediate radioresistance and IR-induced tumour repopulation in vivo [302].

#### The roles of CSC signalling pathways in radioresistance

Several lines of evidence support the assertion that CSCs are implicated in radioresistance [126–129, 303–306]. Clinical studies showed that the expression of CSC markers, including CD44, CD133, and ALDH1, is correlated with a poor prognosis after radiotherapy in patients with lung and larynx cancer [303, 304]. The radioresistance of CSCs is associated with both the intrinsic properties of CSCs (increased DNA repair capability, cell cycle status, upregulated ROS scavengers, inhibited apoptosis, induced autophagy, induced survival pathways) and the adaptive responses of CSCs that are caused by IR and by microenvironmental changes (e.g., changes in endothelial cells, ECM, cytokine levels, NO levels, oxygen levels) [198, 305, 307–315]. As mentioned above, CSCs can exhibit additional metabolic reprogramming in response to cancer treatment, and this can lead to adaptive and acquired resistance [198]. IR can also modify the TME, and these factors affect the IR response of CSCs [305].

In particular, CSCs exhibit several biological features that are responsible for resistance to conventional anti-tumour therapies. CSCs commonly express high levels of genes involved in DNA damage response (ATM, SMC1, CHK1, CHK2, p53) and in DNA DSB repair pathways, including homologous recombination genes (BRCA1, Exo1, Rad51, Rad52) and genes involved in NHEJ (XLF), that contribute to radioresistance [307–311]. In addition, overexpression of stem cell factors, such as ALDH, increases the clonogenic capacity of CSCs and decreases their growth rates, thereby also conferring radioresistance [312].

ROS scavengers are also highly expressed in the CSCs in some tumours, and these protect them from ROS-induced damage [313, 314]. Pharmacological depletion of ROS scavengers decreases the colony-forming ability of CSCs and enhances their radiosensitivity, indicating that ROS levels are involved in CSC radioresistance [313].

In addition, regulation of the apoptosis and survival pathways is involved in CSC radioresistance. CD133^+^ liver CSCs exhibit elevated levels of anti-apoptotic Bcl-2, and show activation of the PI3K and ERK pathways, compared with CD133^-^ cells [314]. Furthermore, autophagy is implicated in CSC radioresistance. IR induces a larger degree of autophagy in CD133^+^ CSCs, with upregulation of the autophagy-related proteins LC3, ATG5, and ATG12, as compared with CD133^-^ cells. Inhibition of autophagy enhances the radiosensitivity of CD133^+^ CSCs, suggesting a role for autophagy in radioresistance [315].

#### The roles of oncogenic metabolism signalling pathways in radioresistance

Metabolic alteration leads to adaptive and acquired resistance to cancer treatment. Accumulating evidence suggests that alterations in cancer cell metabolism are associated with radioresistance [245, 316–329]. Radioresistant cells have been shown to exhibit the Warburg effect, with increased glucose uptake and decreased mitochondrial oxidative phosphorylation to support their growth [245]. Consistent with this observation, mitochondrial respiration-deficient ρ(0) cells are more resistant to radiation than ρ(+) cells [317].

High glucose levels are also known to prevent IR-induced cell death and to promote EMT by increasing levels of the DANGER protein (also known as ITPRIP or ‘inositol 1,4,5-trisphosphate receptor [IP_3_R] interacting protein’), resulting in radioresistance [322]. DANGER is known to bind directly to death-associated protein kinase (DAPK) and disrupts the catalytic activity of DAPK, which mediates anoikis (anchorage-dependent apoptosis). IR increases DAPK activity, which enhances p53 transcriptional activity, which leads to anoikis. High glucose levels upregulate DANGER and inhibit DAPK activity, which prevents anoikis and promotes EMT, thereby increasing radioresistance. Much clinical evidence has supported the assertion that high glucose uptake in a tumour translates to a poor prognosis for the patient [322]. Thus, inhibition of the glycolytic switch could be a promising therapeutic strategy for treating many cancers, by enhancing their radiosensitivity [320, 323–328].

In addition, glutamine metabolism has been shown to play critical role in radioresistance. Glutamate is a precursor for glutathione synthesis, which regulates redox homeostasis and thereby contributes to cellular defense systems. Thus, inhibition of GLS markedly enhances the radiosensitivity of cancer cells, suggesting an important role of glutamine metabolism in radioresistance [329]. Because the same metabolic pathways are required for both proliferating normal cells and proliferating cancer cells, understanding the molecular mechanisms of cancer metabolism opens a new therapeutic window to the development of better and more successful cancer treatments, by enabling the targeting of oncogenic metabolic pathways.

## Conclusions

Many types of therapy are used to treat cancer, including surgery, chemotherapy, and ionizing radiation (IR) therapy. IR is a major therapeutic tool for treating a variety of malignant tumours. However, IR paradoxically also enhances the migration and invasiveness of cancer cells by inducing EMT. IR induces stromal, vascular, and immunological changes in the TME that present additional adverse effects for the cancer patient by promoting tumour recurrence and metastasis. These side effects are also commonly observed after chemotherapy.

Cancer cells that undergo EMT not only exhibit enhanced metastatic ability, but also acquire stemness and metabolic alterations. EMT, CSCs, oncogenic metabolism, and the TME have all been shown to play important roles in determining cancer treatment outcomes. It is now understood that metabolic changes are associated with malignant transformation, tumour invasion, and metastasis. Oncogenic metabolism has been shown to drive the EMT and CSC phenotypes; these changes may cause resistance to radiotherapy and promote tumour recurrence. Supporting this view, dysregulated metabolism is known to have played important roles in the evolution of cell motility. Cells with higher metabolic rates evolve to have increased motility in premalignant neoplasms, and this may enable cells to preadapt for subsequent invasion and metastasis [330].

Thus, targeting CSCs, EMT, and oncogenic metabolic pathways may reduce primary tumour recurrence, prevent invasion, and prevent distant metastasis. For example, inhibition of TGF-β signalling with a selective inhibitor of ALK5 seems to enhance radiosensitivity by preventing EMT, disrupting self-renewal capabilities, blocking the DNA damage response, and increasing apoptosis [331–333]. Blocking Akt with an inhibitor, such as GSK690693, may also prove useful in suppressing IR-induced EMT and increasing radiosensitivity [71]. A dual PI3K/mTOR inhibitor, BEZ235, is also known to enhance the radiosensitivity of prostate cancer cells with reduced EMT/CSC phenotypes [299].

IR can increase ROS production, which can loop back and mediate most of the biological effects of IR itself [12–19]. ROS have been closely associated with tumorigenesis and tumour progression. High levels of ROS trigger cell death by causing irreversible damage to cellular components such as proteins, nucleic acids, and lipids, whereas low levels of ROS have been shown to promote tumour progression via growth, invasion, and metastasis [46–52]. Thus, this review suggests that IR-induced ROS may play important roles in the induction of EMT, CSCs, and oncogenic metabolic pathways as undesired side effects. Notably, cancer cells express high levels of antioxidant proteins to detoxify themselves against ROS [47, 49, 51]. Therefore, use of radiotherapy must include considerations of the unique redox status of the target tumour.

p53 is one of the most important tumour suppressors. It is well known that p53 is activated in response to IR-induced DNA damage; p53 induces growth arrest, apoptosis, or senescence-like, irreversible growth-arrest in cancer cells, and these actions constitute the therapeutic effects of IR [8–11]. A recent study showed that elephants are cancer-resistant, potentially because of their multiple copies (40 alleles) of TP53, compared with the smaller number of copies (2 alleles) in humans. Thus, in response to IR-induced DNA damage, elephant cells exhibit higher rates of apoptotic death than human cells, suggesting a role for tumour suppressor p53 in cancer resistance [334]. In addition, while wild-type p53 is a tumour suppressor, the mutant form of p53 has been shown to represent not just a loss-of-function phenotype of the protein, but also a gain-of-function phenotype in terms of pro-oncogenic activities [335]. Interestingly, a recent study showed an opposite result, in which IR-induced p53 played an important role in the development of lymphomas. After IR, p53 promoted bone marrow cell death; this created a favourable environment for the expansion of tumour-initiating cells in the thymus, by decreasing cell competition from the bone marrow. Through this mechanism, p53 promoted the IR-induced development of lymphoma [336]. Thus, radiotherapy needs to be carefully considered regarding its effects on p53.

This review concludes that IR can induce EMT, CSCs, and oncogenic metabolism in many cancer cells, as a side-effect; several other studies also raise the possibility that IR causes unwanted side effects. Therefore, a better understanding of the mechanisms involved in IR-induced EMT, CSCs, and oncogenic metabolism may help improve the effectiveness of radiotherapy.

Furthermore, after chemotherapy, surviving cells have been shown to display EMT and CSC phenotypes, oncogenic metabolism, and additional metabolic reprogramming. Similar roles for the EMT and CSC phenotypes, and for oncogenic metabolism, have been demonstrated in cancer cell chemoresistance. Chemotherapy is known to induce the EMT and CSC phenotypes [163, 337–342]. EMT leads cancer cells to become quiescent circulating tumour cells (CTCs) that enter the bloodstream. These CTCs are transformed into CSCs that display both the EMT phenotype and chemoresistance. Thus, surviving CSCs repopulate the tumour and cause a relapse [337]. For example, cisplatin-resistant cancer cells are known to display enhanced EMT features and CSC properties, via the activation of the Akt/β-catenin/Snail signalling pathway [341]. Chemotherapy is also known to induce metabolic alterations [343–347]. For example, taxol-resistant breast cancer cells exhibit higher LDHA expression and activity than do taxol-sensitive cells. Inhibition of LDHA can resensitise these resistant cells to taxol, suggesting a role for metabolic alteration in chemoresistance [345]. Furthermore, chemotherapy can induce the reverse Warburg effect [348–351]; chemotherapy drives stromal fibroblasts to become CAFs that subsequently exhibit the glycolytic switch, activating the HIF-1, STAT3, TGF-β, JNK/AP1, and NF-κB pathways. These CAFs, in turn, set up synergistic relationships with adjacent epithelial cancer cells to acquire stemness [350]. Therefore, chemotherapy also causes undesired side effects in cancer cells by inducing EMT, CSCs, and oncogenic metabolic pathways, in a manner similar to IR. In the long term, any therapeutic strategy that affects EMT/CSC/oncogenic metabolic behaviour will require patient-personalized considerations of how to best utilize radiotherapy and chemotherapy.

## Abbreviations

ALK5: TGF-β type I receptor kinase
CAFs: Cancer-associated fibroblasts
COX: Cytochrome C oxidase
CS: Citrate synthase
CSC: Cancer stem cell
CTCs: Circulating tumour cells
CXCL12: C-X-C motif chemokine ligand 12
CXCR4: C-X-C chemokine receptor type 4
DAMP: Damage-associated molecular pattern
DAPK: Death-associated protein kinase
Dlx-2: Distal-less homeobox-2
DSBs: DNA double-strand breaks
ECM: Extracellular matrix
EGF: Epidermal growth factor
EMT: Epithelial-mesenchymal transition
ERK: Extracellular signal-regulated kinase
FASN: Fatty acid synthase
FBP1: Fructose-1,6-bisphosphatase 1
GAPDH: Glyceraldehyde-3-phosphate dehydrogenase
G-CSF: Granulocyte-colony stimulating factor
GLS1: Glutaminase 1
GSK3β: Glycogen synthase kinase3β
HIF-1: Hypoxia-inducible factor-1
IR: Ionizing radiation
LDH: Lactate dehydrogenase
LncRNAs: Long noncoding RNAs
LRP: Lipoprotein receptor-related protein
MAPK: Mitogen-activated protein kinase
MCT: Monocarboxylate transporter
MDSCs: Myeloid-derived suppressor cells
MiRNAs: MicroRNAs
MMP: Matrix metalloproteinase
MTOR: Mammalian target of rapamycin
NAC: N-acetylcysteine
NF-κB: Nuclear factor-kappa B
NHEJ: Non-homologous end-joining
NO: Nitric oxide
OXPHOS: Oxidative phosphorylation
PAI-1: Plasminogen activator inhibitor-1
PAK1: p21-activated kinase 1
PC: Pyruvate carboxylase
PDGFR: Platelet-derived growth factor receptors
PDH: Pyruvate dehydrogenase
PDK: Pyruvate dehydrogenase kinase
PI3K: Phosphatidylinositol 3-kinase
PKM2: Pyruvate kinase M2
PPP: Pentose phosphate pathway
PTEN: Phosphatase and tensin homolog
RNS: Reactive nitrogen species
ROS: Reactive oxygen species
SDHB: Succinate dehydrogenase subunit B
STAT3: Signal transducer and activator of transcription 3
TCA: Tricarboxylic acid
TGF-β: Transforming growth factor-β
TME: Tumour microenvironment
UPA: Urokinase-type plasminogen activator
UV: Ultraviolet
VEGF: Vascular endothelial growth factor
α-SMA: α-smooth muscle actin
